RETRACTED

# NFIL3 Facilitates Neutrophil Autophagy, Neutrophil Extracellular Trap Formation and Inflammation During Gout *via* REDD1-Dependent mTOR Inactivation

**DOI:** 10.3389/fmed.2021.692781

**Published:** 2021-09-30

**Authors:** Honghu Tang, Chunyu Tan, Xue Cao, Yi Liu, Hua Zhao, Yi Liu, Yi Zhao

**Affiliations:** Department of Rheumatology and Immunology, West China Hospital, Sichuan University, Chengdu, China

**Keywords:** gout, NFIL3, REDD1, mTOR pathway, autophagy, extracellular neutrophil traps

## Abstract

Autophagy pathways play an important role in immunity and inflammation *via* pathogen clearance mechanisms mediated by immune cells, such as macrophages and neutrophils. In particular, autophagic activity is essential for the release of neutrophil extracellular traps (NETs), a distinct form of active neutrophil death. The current study set out to elucidate the mechanism of the NFIL3/REDD1/mTOR axis in neutrophil autophagy and NET formation during gout inflammation. Firstly, NFIL3 expression patterns were determined in the peripheral blood neutrophils of gout patients and monosodium urate (MSU)-treated neutrophils. Interactions between NFIL3 and REDD1 were identified. In addition, gain- or loss-of-function approaches were used to manipulate NFIL3 and REDD1 in both MSU-induced neutrophils and mice. The mechanism of NFIL3 in inflammation during gout was evaluated both *in vivo* and *in vitro via* measurement of cell autophagy, NET formation, MPO activity as well as levels of inflammatory factors. NFIL3 was highly-expressed in both peripheral blood neutrophils from gout patients and MSU-treated neutrophils. NFIL3 promoted the transcription of REDD1 by binding to its promoter. REDD1 augmented neutrophil autophagy and NET formation by inhibiting the mTOR pathway. *In vivo* experimental results further confirmed that silencing of NFIL3 reduced the inflammatory injury of acute gouty arthritis mice by inhibiting the neutrophil autophagy and NET formation, which was associated with down-regulation of REDD1 and activation of the mTOR pathway. Taken together, NFIL3 can aggravate the inflammatory reaction of gout by stimulating neutrophil autophagy and NET formation *via* REDD1/mTOR, highlighting NFIL3 as a potential therapeutic target for gout.

## Introduction

Gout is a common chronic disorder caused by the deposition of monosodium urate (MSU) crystals that manifests as an acute, self-limiting inflammatory monoarthritis afflicting the joints of the lower limb (1). Neutrophil autophagy and the resultant formation of extracellular neutrophil traps (NETs), extracellular fibrous structures composed of chromatin and granule constituents of neutrophils, are the hallmarks of gout pathology (2, 3). Meanwhile, the prevalence of gout is much higher in men than women before menopause because of the uricosuric effect of estrogen, which explains why women are more susceptible to gout after menopause (4). Clinically, elevated serum urate concentration (hyperuricemia) is regarded as the major risk factor for MSU crystal deposition and development of gout (5). Despite significant advancements in understanding the pathophysiology of gout and access to effective urate-lowering therapies, treatment of gout remains suboptimal (6).

RETRACTED

Nuclear-factor, interleukin 3 regulated (NFIL3), also known as E4BP4, an important transcription factor in the immune system, has been extensively implicated in the biological function and development of immune-mediated diseases (7). NFIL3 is primarily expressed in DC, T cells, and various other immune cells (8). Moreover, mutations in NFIL3 are known to sensitize the development of arthritis in both mice and humans and rewire the innate immune system for excessive interleukin (IL)-1β production (9). Initial analyses of the JAPSPAR database in the current study predicted the presence of multiple NFIL3 binding domains in the regulated in development and DNA damage responses 1 (REDD1) promoter region. Inherently, REDD1 represents a conserved protein that can be transiently induced upon multiple stimuli, while its expression can potentially serve as an early biomarker for several diseases including inflammatory diseases, neurodegenerative disorders and cancer (10). What's more is that neutrophils exhibit increased expressions of REDD1 following active ulcerative colitis, a chronic inflammatory disease, wherein the increase REDD1 expression induces inflammation, autophagy, and NET release of neutrophils, which is associated with inhibition of the mechanistic target of rapamycin (mTOR) (11). The hard done work of our peers has further revealed that mTOR is an atypical serine/threonine protein kinase of the phosphoinositide 3-kinase (PI3K)-related kinase family, and further implicated in several human diseases due to its regulation on numerous major cellular processes (12). Furthermore, pharmacological inhibition of the mTOR pathway is associated with increased NET release following neutrophil stimulation *via* up-regulation of autophagy (13). In lieu of these findings, we hypothesized that NFIL3 might play a crucial role in gout progression *via* regulation of the REDD1/mTOR axis, and thus performed a series of experiments to investigate the association between NFIL3 and the REDD1/mTOR signaling along with their interactions in gout, aiming to uncover novel therapeutic targets against the disease.

RETRACTED

## Materials and Methods

### Ethics Statement

The current study was approved by the Ethics Committee of West China Hospital, Sichuan University and performed in strict accordance with the *Declaration of Helsinki*. Signed informed consents were obtained from all participants prior to sample collection. Animal experimentation in the current study was approved by the Ethics Committee of West China Hospital, Sichuan University and conformed to the Guide for the Care and Use of Laboratory Animals published by the US National Institutes of Health. Extensive efforts were made to minimize the number and suffering of the experimental animals.

### Microarray-Based Gene Expression Profiling

First, the gout-related gene expression dataset GSE160170 was retrieved from the Gene Expression Omnibus (GEO) database (https://www.ncbi.nlm.nih.gov/geo/), which comprised of six normal samples and six disease samples. Differential analysis was subsequently conducted using the R language “limma” package with |logFC| > 1 and *p* < 0.05 (False discovery rate method was used to correct the difference *p*-value) set as the threshold to obtain the differentially expressed genes (DEGs) in gout. In addition, the transcription factors included in JASPAR were downloaded from the Harmonizome database (https://maayanlab.cloud/Harmonizome/). The interaction of the candidate transcription factors and DDIT4 was analyzed using the GeneMANIA database (http://genemania.org/), with the related genes and interaction scores obtained. The JASPAR database (http://jaspar.genereg.net/) was further employed to predict the binding domain of NFIL3 in the DDIT4 promoter. Finally, the DDIT4-related genes were subjected to Kyoto encyclopedia of genes and genomes (KEGG) enrichment analysis using the KOBAS3.0 database (http://kobas.cbi.pku.edu.cn/kobas3).

### Clinical Sample Collection

Gout patients admitted at the West China Hospital, Sichuan University between March 2019 and March 2020 were included in the current study. These patients met the 1977 American College of Rheumatology classification criteria, presenting with no history of cancer, hematopathy, kidney disease, infection, or other autoimmune diseases. Healthy individuals with matching ages at the same admission time were included as healthy controls. Detailed clinical characteristics are listed in Supplementary Table 1. Blood samples were then collected from gout patients and healthy controls, and the serum was isolated to determine the expression patterns of related inflammatory factors. Simultaneously, neutrophils were isolated for reverse transcription quantitative polymerase chain reaction (RT-qPCR).

### Preparation of MSU Crystals

Initially, 1.0 g of uric acid (Sigma-Aldrich Chemical Company, St Louis, MO, USA) was dissolved in 200 mL of boiling distilled water containing 6.0 mL of 1 M NaOH solution. After the pH value of the solution was adjusted to 7.2 with HCl, the formed crystals were heated and sterilized at 180°C for 2 h. The solution was then stirred at room temperature to cool gradually and stored overnight at 4°C. The following day, the precipitate was filtered from the solution, dried, and suspended in phosphate-buffered saline (PBS) at a concentration of 50 mg/mL. All reagents were prepared without pyrogen.

RETRACTED

### Measurement of Endotoxin in MSU

Pierce limulus amebocyte lysate (LAL) Chromogenic Endotoxin Quantitation kits (Thermo Fisher Scientific Inc., Waltham, Massachusetts, USA) was employed for endotoxin contamination determination. Standard curves were plotted using *Escherichia coli* (*E. coli*) endotoxins at the concentrations of 1, 0.5, 0.25, and 0.1 EU/mL. Endotoxin-free water served as a negative control (NC) and MSU as an unknown sample. The absorbance value of the sample was measured at 405 nm using a microplate reader (Thermo Fisher Scientific).

### Isolation and Culture of Neutrophils

Neutrophils [polymorphonuclear cells (PMNs)] were isolated from the peripheral blood samples of healthy controls. Heparin was added to prevent clotting, and red blood cells were removed using the dextran precipitation method (GE Healthcare, Little Chalfont, Buckinghamshire, UK). The neutrophils were separated by 5-step percoll gradient centrifugation. The autologous serum was prepared by centrifugation and aseptic filtration. The purified neutrophils were then resuspended in Roswell Park Memorial Institute (RPMI) 1640 medium (Gibco Company, Grand Island, NY, USA) and added with 5% of autologous serum to a final concentration of 5 × 10^6^ cells/mL. Wright staining and fluorescence-activated cell sorting (FACS) analysis revealed that the content of monocytes or lymphocytes in the suspension of neutrophils was <0.1%. The survival rate of neutrophils was over 98% after 4 h of culture, as illustrated by trypan blue staining and Annexin-V/propidium iodide FACS analysis. Neutrophils were treated with 250 μg/mL of MSU for 20 h for *in vitro* stimulation.

### Cell Treatment

Adenovirus packaging system, adenovirus over-expression vector (ADV1) and shRNA synthesis adenovirus vector (ADV4) were procured from Shanghai GenePharma Co., Ltd. (Shanghai, China). GenePharma was commissioned to synthesize the adenovirus expressing shRNA (sh)-negative control (NC), sh-NFIL3, sh-REDD1, NFIL3 over-expression (Ad-NFIL3), REDD1 overexpression (Ad-REDD1) and over-expression control (Ad-NC). HEK293T cells were co-transfected with the packaging virus and the target vector. After 48 h of cell culture, the supernatant was collected. Afterwards, the virus particles were filtered from the supernatant following centrifugation after which the virus titer was detected.

RETRACTED

The virus at the logarithmic phase of growth was harvested and the titer was 10^8^ TU/mL. Cells at the logarithmic phase of growth were trypsinized and mechanically dissociated into a cell suspension containing 5 × 10^4^ cells/mL. The cell suspension was then seeded into 6-well plates (2 mL per well), and cultured overnight at 37°C. Next, the cells were treated with sh-NC, sh-NFIL3, Ad-NC, Ad-NFIL3, sh-REDD1, sh-NC + dimethyl sulphoxide (DMSO), sh-REDD1 + DMSO, sh-REDD1 + Rapamycin (mTOR inhibitor; MedChemExpress Company, USA; 100 nM), sh-NC + Ad-NC, sh-NFIL3 + Ad-NC and sh-NFIL3 + Ad-REDD1. After 48 h of infection, the cells were collected for subsequent experimentation.

### Dual-Luciferase Reporter Assay

The REDD1 promoter sequence with the putative NFIL3 binding sites was amplified using PCR, and then cloned into the pGL3 vector (Promega Corporation, Madison, WI, USA), with the pGL3-REDD1 vector plasmid obtained. The over-expression vector of NFIL3 was constructed. Next, the pGL3-REDD1 vector was co-transfected with oe-NFIL3 or oe-NC into HEK-293T cells. After 48 h of culture, the luciferase activity was determined using a Dual Luciferase Reporter Assay kit (D0010, GeneCopoeia, Beijing Solarbio Science & Technology Co., Ltd., Beijing, China) on a Glomax 20/20 luminometer (E5311, Promega, Zhongmei Biotechnology Co., Ltd., Shannxi, China), which was expressed as the ratio of relative luciferase activity of firefly luciferase to that of renilla luciferase.

### NET Formation Assay

PMNs were plated in a 96-well black plate (#3603, Corning Glass Works, Corning, N.Y., USA) coated with poly-L-lysine containing 0.2% Sytox buffer (Life Technologies, Grand Island, NY) at a density of 1 × 10^5^ cells/well. Subsequently, the PMNs were stimulated for 3 h with 250 μg/mL MSU and 100 nM phorbol myristate acetate (PMA; #P8139-10MG, Sigma-Aldrich). To remove background fluorescence, designated wells were treated with DNAse I (#AMPD1-KT, Sigma-Aldrich). Next, 1% of Triton X-100 (#BP151-100, Thermo Fisher Scientific) was added to wells to adjust the DNA staining to 100%. Before the end of assay, the wells were treated with 4 μM Sytox green (#S7020, Life Technologies) to stain the extracellular DNA. Fluorescence was assayed on a fluorescence microplate reader (Varioskan Ascent, Thermo Fisher Scientific) at 37°C for 6 h using an excitation wavelength of 530 nm. To quantify the amount of extracellular DNA (as a percentage of total DNA), the fluorescence intensity of the DNase containing wells from the comparative control was subtracted, and divided by the fluorescence intensity emitted from “PMN + Triton X-100” wells (total DNA present) (14, 15). The normalized fluorescence increase (saponin-treated PMNs) at the maximum was the release of extracellular DNA, expressed as the percentage of the maximum (% max).

RETRACTED

### Immunofluorescence Staining

A total of 2 × 10^5^ PMNs were plated in a 24-well plate on poly-L-lysine coverslips and allowed to equilibrate/adhere for 10 min. Subsequently, the cells were stimulated for 3 h with 200 nM PMA and 100 μg/mL MSU to induce NET formation. Next, the cells were fixed with 10% neutral buffered formalin (#HT501128-4L, Sigma-Aldrich) overnight. The following day, the coverslips were blocked and permeabilized with 5% goat serum and 0.1% Triton X-100 for 1 h. Anti-neutrophil elastase antibody (#ab21595, dilution ratio of 1:200, Abcam Inc., Cambridge, UK) was used to visualize NETs. DNA was then stained with 1 μg/mL 4',6-diamidino-2-phenylindole (DAPI; #D1306, Molecular Probes, Eugene, OR, USA). Goat anti-rabbit Alexa 594 (#R37117, Thermo Fisher Scientific) served as the secondary antibody. Images were captured with the help of a laser scanning confocal fluorescence microscope (Olympus Fluoview FV10i) using a 60 × objective.

### Enzyme-Linked Immunosorbent Assay

Serum samples from gout patients or health controls were collected by centrifugation and stored at −80°C for cytokine assessment. IL-17 (#SEA063Hu) and IL-23 (#SEA384Hu) kits were procured from the USCN Life Science and Technology Company, while IL-1β (#88-7013-88) kits were purchased from eBioscience (San Diego, CA, USA). These kits were also used to measure cytokines in the cell supernatant and mouse serum. The levels of NETs in serum samples were detected using myeloperoxidase-DNA (MPO-DNA) kits. The optical density value of each well was measured with the help of a microplate reader.

### Chromatin Immunoprecipitation

Cells were fixed with 1% formaldehyde for 10 min to produce DNA-protein cross-linking. Subsequently, the cells were lysed with cell lysis buffer (20 mM Tris-HCL, pH 8.0, 85 mM KCL, 0.5% NP40 and protease inhibitor) and centrifuged to obtain the nucleus. The pellet was then subjected to ultrasonic treatment to produce 200–1,000 bp chromatin fragments. Next, the lysate was incubated with antibodies against NFIL3 (11773-1-AP, Proteintech ProteinTech Group, Chicago, IL, USA) and IgG (serving as NC) at 4°C overnight. The DNA that could bind to NFIL3 was sedimented by centrifugation using Pierce protein A/G Magnetic Beads (88803, Thermo Fisher Scientific, San Jose, CA, USA). The obtained sediment was centrifuged at 12,000 × g for 5 min. The non-specific complex was then washed away from the precipitate, followed by de-crosslinking at 65°C overnight. Finally, the precipitated DNA was analyzed using RT-qPCR with the REDD1 primer (forward sequence was 5′-GGCCACGGGGATGAAGCAGA-3′ and reverse sequence was 5′-GCTGAGCTCGCTCTCAAGGGCATCGGTCGA-3′).

RETRACTED

### RT-qPCR

Total RNA content was extracted from the cells using the TRIzol reagent (15596026, Invitrogen Inc., Carlsbad, CA, USA), and then reverse-transcribed into complementary DNA (cDNA) according to the instructions of the PrimeScript RT reagent kit (RR047A, Takara, Japan) at 37°C for 30–50 min and 85°C for 5 s. Subsequently, RT-qPCR was performed using Fast SYBR Green PCR kits (Applied Biosystems Inc. Carlsbad, CA, USA) on the ABI PRISM 7300 RT-qPCR system (Applied Biosystems). Triplicate wells were set for all investigations. The primer sequences are shown in Supplementary Table 2. The fold changes were calculated by means of relative quantification (2^−ΔΔCt^ method) with GADPH serving as the loading control.

### Western Blot Analysis

Total protein content was extracted from the cells using a radioimmunoprecipitation assay (RIPA) lysis buffer (Shanghai Beyotime Biotechnology Co. Ltd., Shanghai, China) containing 1% phenylmethylsulphonyl fluoride (PMSF), with the concentration determined using bicinchoninic acid (BCA) protein assay (Pierce; Thermo Fisher). Next, 50 μg protein was separated using separation gel and concentrated gel and transferred onto polyvinylidene fluoride membranes. The membrane was then blocked with 5% skimmed milk powder for 1 h at room temperature and probed at 4°C overnight with the following diluted primary antibodies: NFIL3 (rabbit, 11773-1-AP, dilution ratio of 1: 2,000, Proteintech), REDD1 (rabbit, 10638-1-AP, dilution ratio of 1: 500, Proteintech), S6 (mouse, #2317, dilution ratio of 1:1,000, Cell Signaling Technology, Beverly, MA, USA), 4EBP1 (rabbit, #9452, dilution ratio of 1:1,000, Cell Signaling Technology), phosphorylated (p)-S6 (rabbit, #4858, dilution ratio of 1: 2,000, Cell Signaling Technology), p-4EBP1 (rabbit, #2855, dilution ratio of 1: 1,000, Cell Signaling Technology), LC3 (rabbit, #4108, dilution ratio of 1:1,000, Cell Signaling Technology) and β-actin (mouse, AC004, dilution ratio of 1:10,000, ABclonal, China, serving as lading control). Following 3 rinses with PBST, the membrane was re-probed with the horseradish peroxidase-labeled secondary antibody goat anti-mouse or goat anti-rabbit (dilution ratio of 1:10,000, Boster Biological Technology Co., Ltd., Wuhan, Hubei, China) for 1 h at room temperature. Afterwards, the bands were visualized using enhanced chemiluminescence (Thermo Fisher Scientific) and band intensities were quantified using the Image J software.

RETRACTED

### Acute Gouty Arthritis Mouse Model Establishment and Animal Treatment

A total of 50 male C57BL/6 mice (weighing 18–22 g, aged 6 weeks; Hunan SJA Laboratory Animal Co., Ltd., Human, China) were housed at 25–27°C and 45–50% humidity with a 12-h light/dark cycle for 1 week. The mice were fasted for 12 h before administration, and given *ad libitum* access to drinking water at other times.

The mice were intraperitoneally anesthetized with 10 mg/kg ketamine, and then administered with PBS, MSU, MSU + sh-NC + Ad-NC, MSU + sh-NFIL3 + Ad-NC and MSU + sh-NFIL3 + Ad-REDD1 (n = 10). The adenovirus (10 μL of each, 1.2 × 10^9^ vg/mL) was then injected into the joint cavity of mice. The MSU mice were injected with 1 mg MSU crystal (1 mg MSU dissolved in 40 μL PBS) into the hind ankle joint using a Hamilton syringe. Meanwhile, the PBS-treated mice were injected with same volumes of sterile PBS into the hind ankle joint to serve as the control. After 24 h, the swelling of ankle joint was measured with electronic calipers, and blood samples were obtained through an axillary vascular incision of right subclavian vein during euthanasia. Afterwards, the serum was isolated for subsequent experimentation. The ankle joint tissues were collected, fixed with 10% paraformaldehyde in PBS, decalcified for 10 days and embedded in paraffin for histological analysis. The obtained paraffin sections were stained with hematoxylin and eosin (HE) for routine morphological evaluation.

### Cytokine Analysis and MPO Activity Detection

The serum was collected for cytokine measurement with the help of ELISA kits. The hind ankle was separated and cut in half. One half was used for histological analysis, and the other was placed in RIPA or TRIzol reagent. The supernatant was subsequently collected by centrifugation after lysis to detect the MPO activity. Neutrophils were isolated using the same method as those from human peripheral blood samples to detect the expression patterns of related proteins and RNA. MPO activity in human peripheral blood neutrophils can be used as a quantitative detection method for neutrophil separation, that is, a colorimetric assay kit (Nanjing Jiancheng Bioengineering Institute, Nanjing, China) was used to determine MPO activity in joint tissues.

### Statistical Analysis

Statistical analyses were performed using the SPSS 22.0 statistical software (IBM Corp. Armonk, NY, USA) and GraphPad Prism 7.0 software. Measurement data were summarized by mean ± standard deviation. Data between two groups were analyzed using unpaired *t*-test, while data among multiple groups were assessed using one-way analysis of variance (ANOVA). Analysis of homogeneity of variance was confirmed by Levene's test where data obeying homogeneity of variance were compared with Dunnett's *t*-test and LSD-*t*-test, while data with defect variances were compared by Dunnett's T3. A value of *p* < 0.05 was considered statistically significant.

RETRACTED

## Results

### NFIL3 Is Highly-Expressed in Neutrophils of Peripheral Blood of Gout Patients and MSU-Treated Neutrophils

Initially, differential analyses of the GSE160170 dataset revealed a total of 887 DEGs related to gout (Figure 1A). Subsequent intersection analysis of these genes and transcription factors included in the JASPAR (Figure 1B) showed that seven transcription factors were significantly differentially expressed in the GSE160170 dataset (Figure 1C). Moreover, detection of the differential expressions of the seven transcription factors in the dataset revealed that NFIL3 exhibited the most significant expression (Supplementary Table 3). In addition, the results of RT-qPCR and Western blot analysis showed that the mRNA and protein expression levels of NFIL3 were higher in peripheral blood neutrophils of gout patients than those of healthy controls (Figures 1D,E). Meanwhile, NFIL3 mRNA and protein expression levels were also found to be increased in MSU-treated neutrophils compared with PBS-treated neutrophils (Figures 1F,G). Together, these findings indicated that NFIL3 was abundantly expressed in both peripheral blood neutrophils of gout patients and MSU-treated neutrophils.

**Figure 1:** NFIL3 is amplified in the peripheral blood neutrophils of gout patients and MSU-treated neutrophils. **(A)** A heat plot of differential mRNA expression in the GSE160170 dataset. The abscissa represents the –log10 *p*-value and ordinate represents the logFC; the red dots indicate highly expressed genes in diseases, and the green dots indicate weakly expressed genes. **(B)** Venn diagram analysis of differential mRNAs and transcription factors included in the JASPAR. The central represents the intersection of two groups of data. **(C)** A heat plot of differential transcription factors in the GSE160170 dataset. The abscissa represents the sample number and the ordinate represents the gene name; the upper dendrogram shows the sample clustering and the histogram at the upper left refers to color gradation. **(D)** mRNA expression of NFIL3 determined by RT-qPCR in the peripheral blood neutrophils of 28 gout patients and 20 healthy controls. ***p < 0.01, compared to healthy controls. **(E)** Western blot analysis of NFIL3 protein in the peripheral blood neutrophils of 28 gout patients and 20 healthy controls. ***p < 0.001, compared to healthy controls. **(F)** mRNA expression of NFIL3 determined by RT-qPCR in MSU-treated neutrophils. ***p < 0.001, compared to PBS-treated neutrophils. **(G)** Western blot analysis of NFIL3 protein in MSU-treated neutrophils. ***p < 0.001, compared to PBS-treated neutrophils. Data are shown as mean ± standard deviation of three technical replicates. Data between two groups were compared using unpaired *t*-test.

RETRACTED

### NFIL3 Promotes the Transcription of REDD1 While NFIL3 Silencing Represses Its Expression

We further aimed to determine the downstream target of NFIL3 in gout. The JAPSPAR database predicted the presence of multiple NFIL3 binding domains in the REDD1 promoter region (Supplementary Table 4). Meanwhile, RT-qPCR and Western blot analysis results demonstrated higher REDD1 mRNA and protein expression levels in peripheral blood neutrophils of gout patients than those of healthy controls (Figures 2A,B). Similarly, the mRNA and protein expression levels of REDD1 were augmented in MSU-treated neutrophils (Figures 2C,D).

**Figure 2:** NFIL3 promotes the transcription of REDD1. **(A)** mRNA expression of REDD1 determined by RT-qPCR in the peripheral blood neutrophils of 28 gout patients and 20 healthy controls. ***p < 0.001, compared to healthy controls. **(B)** Western blot analysis of REDD1 protein in the peripheral blood neutrophils of 28 gout patients and 20 healthy controls. ***p < 0.001, compared to healthy controls. **(C)** mRNA expression of REDD1 determined by RT-qPCR in MSU-treated neutrophils. **p < 0.01, compared to PBS-treated neutrophils. **(D)** Western blot analysis of REDD1 protein in MSU-treated neutrophils. **p < 0.01, compared to PBS-treated neutrophils. **(E)** The enrichment of NFIL3 in the REDD1 promoter region detected by ChIP assay. **p < 0.01, compared to IgG antibody. **(F)** A schematic diagram of NFIL3 binding sites in the REDD1 promoter region. **(G)** Binding of NFIL3 to the REDD1 promoter analyzed by dual-luciferase reporter assay. ***p < 0.001, compared to cells treated with pGL3-REDD1 + oe-NC. **(H)** mRNA expression of NFIL3 and REDD1 determined by RT-qPCR in neutrophils following NFIL3 silencing or overexpression. **p < 0.01 or ***p < 0.001, compared to cells treated with sh-NC. ###*p* < 0.001, compared to cells treated with Ad-NC. **(I)** Western blot analysis of NFIL3 and REDD1 proteins in neutrophils following NFIL3 silencing or overexpression. **p < 0.01 or ***p < 0.001, compared to cells treated with sh-NC. ##*p* < 0.01 or ###*p* < 0.001, compared to cells treated with Ad-NC. Data are shown as mean ± standard deviation of three technical replicates. Data between two groups were compared using unpaired *t*-test while those among multiple groups were assessed by one-way ANOVA.

RETRACTED

Furthermore, the results of ChIP assay exhibited that NFIL3 was enriched in the REDD1 promoter region (Figure 2E). In addition, dual-luciferase reporter assay further demonstrated that NFIL3 could bind to the REDD1 promoter (Figures 2F,G). Subsequently, the mRNA expression patterns of NFIL3 and REDD1 were determined by RT-qPCR, which revealed a downward trend in MSU-treated neutrophils treated with sh-NFIL3, while increased NFIL3 and REDD1 mRNA expression levels were observed following NFIL3 over-expression (Figure 2H). As shown in Figure 2I, similar findings were also documented in terms of NFIL3 and REDD1 protein levels. Altogether, these findings showed that NFIL3 could facilitate the transcription of REDD1, while knockdown of NFIL3 led to suppression of REDD1 expression.

### REDD1 Promotes Neutrophil Autophagy and Production of Inflammatory Factors Through Inhibition of the mTOR Pathway

To elucidate the role of REDD1 in the progression of gout, we retrieved the REDD1-related genes in the GeneMANIA database (Figure 3A), and the obtained genes were subjected to KEGG enrichment analysis. Subsequent results showed that REDD1-related genes were primarily enriched in the PI3K/AKT, AMPK, mTOR, and autophagy signaling pathways, wherein PI3K/AKT and AMPK were the upstream regulatory factors of mTOR (Figure 3B). Meanwhile, REDD1 is a well-established inhibitor of mTORC1 (16). Therefore, we determined the phosphorylation levels of two downstream effectors of mTORC1 (S6 and 4EBP) by means of Western blot analysis, which revealed a decline in the S6 and 4EBP phosphorylation levels in the peripheral blood neutrophils of gout patients (Figure 3C). Meanwhile, ELISA results showed that the levels of IL-17, IL-23 and IL-1b were all augmented in the peripheral blood of gout patients (Figure 3D). Also, S6 and 4EBP phosphorylation levels were diminished in MSU-treated neutrophils (Figure 3E), and the MSU-treated cell supernatant exhibited increased levels of IL-17, IL-23 and IL-1b (Figure 3F). On the other hand, the mRNA and protein expression of REDD1 were decreased, while S6 and 4EBP phosphorylation levels were enhanced in neutrophils as a result of REDD1 silencing. Furthermore, autophagy related protein LC3 II expression levels were noted to be decreased in neutrophils treated with sh-REDD1 (Figures 3G,H). These findings suggested that silencing of REDD1 could activate the mTOR pathway and inhibit neutrophil autophagy.

**Figure 3:** REDD1 inactivates the mTOR pathway to trigger neutrophil autophagy and inflammatory response. **(A)** REDD1-related genes analyzed by the GeneMANIA database. Each circle in the figure represents a gene, and the line between circles indicates interaction between two genes. **(B)** KEGG enrichment analysis of REDD1-related genes. The abscissa represents GeneRatio, the ordinate represents the entry identifier, the color represents enrichment *p*-value, and the size represents the number of enriched genes in the identifier. **(C)** Western blot analysis of p-S6 and p-4EBP in the peripheral blood neutrophils of 28 gout patients and 20 healthy controls. **(D)** Levels of IL-17, IL-23 and IL-1β in the peripheral blood of 28 gout patients and 20 healthy controls measured by ELISA. **(E)** Western blot analysis of p-S6 and p-4EBP in the MSU-treated neutrophils. **(F)** Levels of IL-17, IL-23 and IL-1β in the MSU-treated cell supernatant measured by ELISA. **(G)** mRNA expression of REDD1 determined by RT-qPCR in neutrophils treated with sh-REDD1. **(H)** Western blot analysis of p-S6, p-4EBP and LC3 II in neutrophils treated with sh-REDD1. **(I)** mRNA expression of REDD1 determined by RT-qPCR in neutrophils treated with sh-REDD1 or combined with Rapamycin. **(J)** Western blot analysis of p-S6, p-4EBP and LC3 II in neutrophils treated with sh-REDD1 or combined with Rapamycin. **(K)** Levels of IL-17, IL-23 and IL-1β in the supernatant of cells treated with sh-REDD1 or combined with Rapamycin measured by ELISA. In **(C,D)**, ***p < 0.001, compared to healthy controls. In **(E,F)**, **p < 0.01, compared to cells treated with PBS; ***p < 0.001, compared to cells treated with PBS. In **(G,H)**, **p < 0.01, compared to cells treated with sh-NC; ***p < 0.001, compared to cells treated with sh-NC. In **(I–K)**, **p < 0.01, compared to cells treated with sh-NC + DMSO; ##*p* < 0.01, compared to cells treated with sh-REDD1 + DMSO; ###*p* < 0.001, compared to cells treated with sh-REDD1 + DMSO. Data are shown as mean ± standard deviation of three technical replicates. Data between two groups were compared using unpaired *t*-test while those among multiple groups were assessed by one-way ANOVA.

RETRACTED

Furthermore, the results of RT-qPCR and Western blot analysis showed that combined treatment with sh-REDD1 and Rapamycin reversed the effect of individual sh-REDD1 treatment on the S6 and 4EBP phosphorylation levels and LC3 II expression (Figures 3I,J). Moreover, ELISA results demonstrated that the levels of IL-17, IL-23 and IL-1β were all diminished in the cell supernatant upon REDD1 silencing, whereas opposite trends were observed upon further treatment with Rapamycina (Figure 3K). Together, these findings indicated that REDD1 could stimulate neutrophil autophagy and induce inflammatory response by disrupting the mTOR pathway.

### REDD1 Promotes the Formation of NETs by Inducing Neutrophil Autophagy

Gout patients are known to exhibit elevated levels of NETs and neutrophil activation markers compared to healthy controls (17). Meanwhile, the REDD1/autophagy pathway possesses the ability to regulate the formation of NETs in human systemic lupus erythematosus (18). Consequently, we speculated that REDD1/autophagy pathway may affect the formation of NETs in gout. For verification, we performed ELISA to detect the levels of NETs in patients with gout and healthy controls, which revealed that the levels of NETs were significantly higher in the peripheral blood of gout patients than those of healthy controls (Figure 4A). Meanwhile, the results of immunofluorescence illustrated that the formation of NETs was enhanced after MSU treatment (Figure 4B).

**Figure 4:** REDD1 induces the formation of NETs by promoting neutrophil autophagy. **(A)** Levels of NETs in the peripheral blood of 28 gout patients and 20 healthy controls measured by ELISA. ***p < 0.001, compared to healthy controls. **(B)** Immunofluorescence staining analysis of the formation of NETs in MSU-treated neutrophils, scale bar = 50 μm. Neutrophil elastase (NE) and DAPI (DNA) were used to stain the cells. The white arrow represents the formed NETs. ***p < 0.001, compared to PBS-treated neutrophils. **(C)** Western blot analysis of LC3 II protein in MSU-induced neutrophils treated with Baf A1. **p < 0.001, compared to MSU-treated neutrophils. **(D)** Immunofluorescence staining analysis of the formation of NETs in MSU-induced neutrophils treated with Baf A1. **p < 0.01, compared to MSU-treated neutrophils. **(E)** Immunofluorescence staining analysis of the formation of NETs in neutrophils treated with sh-REDD1 or combined with Rapamycin, scale bar = 50 μm. **p < 0.01, compared to neutrophils treated with sh-NC and DMSO. ##*p* < 0.01, compared to neutrophils treated with sh-REDD1 and DMSO. Data are shown as mean ± standard deviation of three technical replicates. Data between two groups were compared using unpaired *t*-test while those among multiple groups were assessed by one-way ANOVA.

Subsequent results from Western blot analysis showed that Bafilomycin A1 (Baf A1; an inhibitor of autophagy; MedChemExpress Company, USA; 100 nM, 30 min) could down-regulate the LC3 II protein expression in MSU-treated neutrophils (Figure 4C). In addition, the formation of NETs was retarded following Baf A1 treatment, as revealed by immunofluorescence (Figure 4D). Moreover, silencing of REDD1 could also inhibit the formation of NETs, while this effect could be abrogated by dual treatment with sh-REDD1 and Rapamycin (Figure 4E). Overall, these findings suggested that neutrophil autophagy could promote the formation of NETs, and that REDD1 facilitated the formation of NETs by inducing neutrophil autophagy.

RETRACTED

### Silencing of NFIL3 Suppresses Neutrophil Autophagy and NET Formation by Down-Regulating REDD1 Expression

Furthermore, we elucidated whether NFIL3 affected neutrophil autophagy and the formation of NETs by regulating REDD1 expression. The results of RT-qPCR and Western blot analysis showed that the mRNA and protein expression levels of NFIL3 and REDD1 along with LC3 II protein expressions were all decreased, but S6 and 4EBP phosphorylation levels were increased in neutrophils as a result of NFIL3 silencing; however, further REDD1 over-expression abrogated the effect of NFIL3 silencing (Figures 5A–D; Supplementary Figures 1A–C). Meanwhile, quantitative analysis of NET formation indicated a reduction in NET formation in the absence of NFIL3, whereas additional REDD1 over-expression promoted NET formation (Figure 5E). Cumulatively, these findings NFIL3 silencing could inhibit neutrophil autophagy and NET formation by reducing the expression of REDD1.

**Figure 5:** NFIL3 silencing contributes to suppressed neutrophil autophagy and NET formation, which is related to downregulated expression of REDD1. **(A)** mRNA expression of NFIL3 and REDD1 determined by RT-qPCR in neutrophils treated with sh-NFIL3 or combined with Ad-REDD1. **(B)** Western blot analysis of NFIL3 and REDD1 proteins in neutrophils treated with sh-NFIL3 or combined with Ad-REDD1. **(C)** Western blot analysis of p-S6 and p-4EBP1 in neutrophils treated with sh-NFIL3 or combined with Ad-REDD1. **(D)** Western blot analysis of LC3 II protein in neutrophils treated with sh-NFIL3 or combined with Ad-REDD1. **(E)** NET formation in neutrophils treated with sh-NFIL3 or combined with Ad-REDD1, scale bar = 50 μm. ***p < 0.001, compared to neutrophils treated with sh-NC + Ad-NC. ##*p* < 0.01, compared to neutrophils treated with sh-NFIL3 + Ad-NC. ###*p* < 0.001, compared to neutrophils treated with sh-NFIL3 + Ad-NC. Data are shown as mean ± standard deviation of three technical replicates. Data among multiple groups were assessed by one-way ANOVA.

### Silencing of NFIL3 Represses Neutrophil Autophagy and NET Formation, Thus Alleviating the Inflammatory Injury in Mice With Acute Gouty Arthritis *via* the REDD1/mTOR Axis

Lastly, we proceeded to verify whether silencing NFIL3 could regulate the REDD1/mTOR axis to inhibit neutrophil autophagy and NET formation, thereby affecting the inflammatory injury in mice with acute gouty arthritis. Observational results illustrated that the ankles of MSU-induced mouse model of acute gouty arthritis were swollen compared to control mice. HE staining was further performed to determine the pathological changes in the tissues, which revealed that silencing of NFIL3 reduced the ankle swelling of mice, while further REDD1 over-expression increased the ankle swelling (Figures 6A,B).

RETRACTED

**Figure 6:** NFIL3 silencing impairs neutrophil autophagy, reduces NET formation and inflammatory injury in mice with acute gouty arthritis *via* the REDD1/mTOR axis. PBS-treated mice served as the control and MSU mice were treated with sh-NFIL3 or combined with Ad-REDD1. **(A)** Representative microscopic views of ankle joint swelling of mice (the left), and the corresponding quantitative analysis (the right). **(B)** The representative images of pathological changes in the joint tissues of mice following HE staining, scale bar = 25 μm. **(C)** mRNA expression of NFIL3 determined by RT-qPCR in the neutrophils of the joint tissue of mice. **(D)** mRNA expression of REDD1 determined by RT-qPCR in the neutrophils of the joint tissue of mice. **(E)** Western blot analysis of NFIL3 expression in the neutrophils of the joint tissues of mice. **(F)** Quantitative analysis of REDD1 protein expression. **(G)** Quantitative analysis of S6 and 4EBP phosphorylation levels. **(H)** Quantitative analysis of LC3 II protein expression. **(I)** MPO activity in the joint tissue of mice. **(J)** IL-17 levels measured by ELISA in the serum of mice. **(K)** IL-23 levels measured by ELISA in the serum of mice. **(L)** IL-1β levels measured by ELISA in the serum of mice. **(M)** Quantitative analysis of NET formation in the joint tissue of mice. ***p < 0.001, compared to PBS-treated mice. ##*p* < 0.01, compared to MSU mice treated with sh-NC + Ad-NC. ###*p* < 0.001, compared to MSU mice treated with sh-NC + Ad-NC. &, && or &&& *p* < 0.05, compared to MSU mice treated with sh-NFIL3 + Ad-NC. Data are shown as mean ± standard deviation of three technical replicates. Data among multiple groups were assessed by one-way ANOVA. *n* = 10 for mice in each group.

In addition, the results of RT-qPCR and Western blot analysis showed an upward trend in the mRNA and protein expression levels of NFIL3 and REDD1 along with LC3 II protein expressions, while S6 and 4EBP phosphorylation levels were decreased in joint tissues of mice in response to MSU administration (Figures 6C–H, Supplementary Figures 2A–D). On the other hand, mRNA and protein expression levels of NFIL3 and REDD1 along with LC3 II protein expressions were all down-regulated, while S6 and 4EBP phosphorylation levels were up-regulated in joint tissues of mice as a result of NFIL3 silencing. In contrast, combined treatment with sh-NFIL3 and Ad-REDD1 brought about the opposite results.

RETRACTED

As shown in Figure 6I, MSU mice presented with increased MPO activity, which was decreased upon NFIL3 silencing. Conversely, additional REDD1 over-expression augmented the MPO activity. Meanwhile, the results of ELISA displayed increased levels of IL-17, IL-23, IL-1β and NETs in the serum of MSU mice, whereas opposite trends were observed following NFIL3 silencing. In addition, combined treatment with sh-NFIL3 and Ad-REDD1 contributed to higher levels of IL-17, IL-23, IL-1β and NETs compared to individual sh-NFIL3 treatment (Figures 6J–M). Together, these findings supported that silencing NFIL3 decreased the expression of REDD1 and activated the mTOR pathway, leading to inhibited neutrophil autophagy and NET formation, consequently reducing the inflammatory injury in mice with acute gouty arthritis.

## Discussion

Gout is characterized by severe articular inflammation and pain induced by MSU deposition precipitated by activation of transcription factors (19, 20). Pre-experimentation and confirmation findings in our study demonstrated that transcription factor NFIL3 promoted the transcription of REDD1, induced a subsequent inhibition of mTOR pathway, and enhanced the neutrophil autophagy and NET formation, consequently preventing the inflammatory response of gout.

Initial findings in our study revealed that NFIL3 was highly-expressed in the neutrophils of peripheral blood of gout patients and MSU-treated neutrophils. Patients with systemic lupus erythematosus, an autoimmune disease, are also known to exhibit increased expressions of NFIL3, which were further positively-correlated with disease activity (21). Similarly, another study documented up-regulated levels of NFIL3 in osteosarcoma tissues, such that these levels promoted the proliferation, migration, and invasion of osteosarcoma cells (22). Meanwhile, NFIL3 was recently indicated to exacerbate lung cancer cell migration and invasion of lung cancer cells in a PrPc-dependent manner (23), while another study demonstrated that NFIL3 exerts function on chromatin to alter cancer cell behavior in the regulation of FOXO-triggered gene expression in cancer (24). From an inflammation perspective, NFIL3 is known to serve as an important transcription factor of the immune system, wherein NFIL3 silencing can down-regulate the pro-inflammatory cytokine IL-16 (25). On the other hand, NFIL3 is capable of up-regulating Tim-3 and IL-10 expression as well as T-cell dysfunction (26).

Furthermore, NFIL3 is known to possess the ability to serve as a transcriptional activator for several genes, such as PRNP and IGF2R, by virtue of direct-binding to their promoter regions (23, 27). In accordance with this ability, our findings uncovered that NFIL3 promoted the transcription of the REDD1 gene by binding to its promoter region. REDD1 is aberrantly up-regulated in neutrophils during disease attacks, whereas during times of adrenergic stress, REDD1-induced autophagy can trigger a pyrin-driven IL-1β maturation and the release of IL-1β-bearing NETs (28). Meanwhile, augmentation of neutrophil autophagy can drive excessive NET production, leading to the resultant thromboinflammation during systemic lupus erythematosus, which were previously correlated with up-regulated expressions of REDD1 (18). Concurrently, these findings reflect that neutrophil autophagy can promote the formation of NETs, and that REDD1 facilitated the formation of NETs by inducing neutrophil autophagy. It is also noteworthy that elevated levels of NETs and neutrophil activation markers have been detected in gout patients relative to healthy controls (17). Therefore, inhibiting the NFIL3/REDD1 axis could provide novel therapeutic approaches against neutrophil autophagy, NET formation and inflammatory response in gout.

RETRACTED

Moreover, subsequent experimentation in our study revealed that REDD1 inactivated the mTOR pathway to trigger neutrophil autophagy, neutrophil autophagy, and inflammatory response. Consistently, REDD1 is known to exhibit adverse correlation with the mTOR pathway, as evidenced by inhibition of iron chelation-induced mTORC1 due to activation of REDD1 (29). In addition, REDD1 over-expression can lead to inhibition of the phosphorylation of mTOR and its downstream effectors P70/S6 kinase and 4EBP1 (30). Importantly, another study illustrated that promoted neutrophil autophagy as well as up-regulation of autophagy-related proteins LC3B, Dynein and Beclin-1 were attributed to decreased expressions of mTOR (31). Furthermore, mTOR pathway inhibition was suggested to contribute to NET formation and NET-induced thromboinflammation (32). However, one recent study performed by Nadia Vazirpanah et, al. documented activation of the mTOR signaling pathway in PBMC (33), which is not consistent with our findings. This can be attributed to the usage of Ficoll density gradient centrifugation to extract PBMCs, which did not contain neutrophils. What's more, gouty arthritis is attributed to acute inflammation characterized by the recruitment of macrophages and MSU crystal deposition-induced neutrophils in the joints (34). In our study, we isolated and treated neutrophils with MSU to establish an *in vitro* model, while MSU crystals were injected to construct a mouse model of acute gouty arthritis. Expectedly, NFIL3 was found to be highly-expressed in neutrophils treated with MSU. Meanwhile, the results of *in vitro* cell experimentation revealed that NFIL3 could transcriptionally activate REDD1, while silencing of NFIL3 inhibited the expression of REDD1 in neutrophils. Furthermore, REDD1 was validated to promote neutrophil autophagy and NET formation by inhibiting the mTOR pathway. Cumulatively, it could be inferred that NFIL3 could potentially accelerate neutrophil autophagy and NET formation, thus stimulating the inflammatory injury during the progression of acute gouty arthritis *via* REDD1-mediated mTOR inactivation. The underlying relationship between NFIL3 and mTOR requires further investigation due to the lack of available literature.

RETRACTED

## Conclusion

To summarize, the current study illustrated a novel pathogenic mechanism that critically implicates the NFIL3/REDD1/mTOR signaling in neutrophil autophagy, NET formation and the resultant inflammatory response following gout (Figure 7). Translating these findings into new diagnostic or therapeutic strategies may be beneficial to patients afflicted by gout and its complications, thus constituting a future challenge.

**Figure 7:** Schematic diagram of the mechanism by which NFIL3 affects gout. NFIL3 promotes the transcription of REDD1 and inhibits the mTOR pathway, thus activating the autophagy of neutrophils and inducing the formation of NETs, eventually aggravating the inflammatory response of gout.

## Data Availability Statement

The original contributions presented in the study are included in the article/Supplementary Material, further inquiries can be directed to the corresponding author/s.

## Ethics Statement

The studies involving human participants were reviewed and approved by West China Hospital, Sichuan University. The patients/participants provided their written informed consent to participate in this study. The animal study was reviewed and approved by West China Hospital, Sichuan University.

## Author Contributions

HT conceived and designed research. CT performed experiments. XC interpreted results of experiments. YL (fourth author) analyzed data. HZ prepared figures. YL (sixth author) drafted paper. YZ edited and revised manuscript. All authors contributed to the article and approved the submitted version.

## Funding

This study was supported by National Natural Science Foundation of China (81771742, 81273286); Project of Sichuan Medical Association (JH20180101) and Project of Sichuan Provincial Department of Health (JH20150441).

## Conflict of Interest

The authors declare that the research was conducted in the absence of any commercial or financial relationships that could be construed as a potential conflict of interest.

RETRACTED

## Publisher's Note

All claims expressed in this article are solely those of the authors and do not necessarily represent those of their affiliated organizations, or those of the publisher, the editors and the reviewers. Any product that may be evaluated in this article, or claim that may be made by its manufacturer, is not guaranteed or endorsed by the publisher.

## Supplementary Material

Supplementary Figure 1 Representative images of western blot analysis in Figure 5. **(A)** Western blot protein band of NFIL3 and REDD1 proteins in neutrophils treated with sh-NFIL3 or combined with Ad-REDD1. **(B)** Western blot protein band of p-S6 and p-4EBP1 in neutrophils treated with sh-NFIL3 or combined with Ad-REDD1. **(C)** Western blot protein band of LC3 II protein in neutrophils treated with sh-NFIL3 or combined with Ad-REDD1.

Supplementary Figure 2 Representative images of western blot analysis in Figure 6. **(A)** Western protein band of NFIL3 in the neutrophils of the joint tissues of mice. **(B)** Western blot protein band of REDD1 in the neutrophils of the joint tissues of mice. **(C)** Western blot protein band of S6, 4EBP1, p-S6, and p-4EBP1 protein expression. **(D)** Western blot protein band of LC3 I and LC3 II protein expression.

Supplementary Table 1 Clinical characteristics of gout patients and healthy controls.

Supplementary Table 2 Primer sequences for reverse transcription quantitative polymerase chain reaction.

Supplementary Table 3 The differential expression of the seven transcription factors in the dataset.

Supplementary Table 4 Prediction result of the JAPSPAR database.
